The article "Analysis of the Application Effect of Exercise Rehabilitation Therapy Based on Data Mining in the Prevention and Treatment of Knee Osteoarthritis" was published in 2022. Journal: Comput Math Methods Med.

# Analysis of the Application Effect of Exercise Rehabilitation Therapy Based on Data Mining in the Prevention and Treatment of Knee Osteoarthritis

**DOI:** 10.1155/2022/2109528

**Published:** 2022-09-05

**Authors:** Wei Liu, Congan Wang, Gongchang Yu, Bin Shi, Jingwen Wang

**Affiliations:** ^1^Department of Public Health, Neck-Shoulder and Lumbocrural Pain Hospital of Shandong First Medical University, Jinan, Shandong 250062, China; ^2^School of Graduate Education, Shandong Institute of P.E. and Sports, Jinan, Shandong 250100, China

## Abstract

**Objective:**

To analyze the application effect of exercise rehabilitation therapy based on data mining in the prevention and treatment of knee osteoarthritis.

**Methods:**

Based on clinical data mining technology, that is, using complex network technology and association rules, the medical records of 1612 patients with KOA in the Department of Rheumatology and Immunology of our hospital were retrospectively analyzed, and they were divided into groups according to whether they used exercise rehabilitation therapy (*n* = 786), and the control treatment group (*n* = 826), the curative effect, the improvement of inflammatory factors and immune factors, the visual analogue scale (VAS), the knee joint function score (Lysholm), and the quality of life (WOMAC) scale were compared between the two groups score, analyze the relationship between VAS and Lysholm score and prognosis quality of life, and compare the recurrence within 12 months between the two groups.

**Results:**

The data mining results showed that the curative effect of the exercise rehabilitation therapy group was significantly higher than that of the control treatment group (*P* < 0.05); the improvement of VAS and Lysholm scores of the exercise rehabilitation therapy group was significantly better than that of the control treatment group (*P* < 0.05). The improvement effect of inflammatory indexes and immune cytokines was significantly better than that of the control treatment group (*P* < 0.05); the improvement of WOMAC in the exercise rehabilitation therapy group was significantly better than that of the control treatment group (*P* < 0.05); VAS and WOMAC scores were significantly positively correlated (*r* = 0.579, *P* < 0.05); Lysholm score was positively correlated with WOMAC score (*r* = −0.563, *P* < 0.05); the recurrence rate of exercise rehabilitation therapy group was 5.09%, which was significantly lower than that of control treatment group (17.63% (*χ*^2^ = 11.967), *P* < 0.05).

**Conclusion:**

Exercise rehabilitation therapy for KOA patients can effectively improve inflammatory and immune factors in patients, enhance knee joint function and prognosis quality of life, and reduce readmission rate, which is worthy of clinical application.

## 1. Background

The main contradiction facing medical treatment in China is that the current medical service capacity cannot meet people's increasing service demand, and the gap between supply and demand is very significant. In terms of demand, with the development of social economy, aging of population, and changes of disease spectrum, the demand for medical services increases, and problems such as insufficient overall health resources, concentration of high-quality medical resources, and imbalance between supply and demand still exist in China [1]. In recent years, artificial intelligence technology has been widely applied in disease prediction, diagnosis, and treatment, drug research and development and other medical and health fields, which has significantly improved the level of medical services, effectively alleviated the above problems, and promoted the healthy development of medical reform policies [2]. Osteoarthritis (OA) is a common joint disease obviously related to aging. Its clinical characteristics are erosion of articular cartilage, subchondral sclerosis, marginal osteophytic hyperplasia (osteophyte formation), and many biochemical and morphological changes of synovial membrane and joint capsule, among which the knee joint is most commonly affected. Knee osteoarthritis (KOA) is easy to form [3]. Clinically, the main manifestations are chronic joint pain, stiffness, swelling, and joint dysfunction. Knee joint is the most complex joint in the human body, and the joint with the largest load and shear force, which is also the main reason for the high incidence of OA in this part [4]. The incidence of OA increases with the increase of age. Therefore, with the aging of the world's population, osteoarthritis is an increasingly serious health problem [5]. In recent years, some healthy therapies have gradually become popular, such as exercise therapy, which can make patients combine muscles and bones, the whole and the local, with remarkable efficacy [6]. The role of sports rehabilitation therapy is the most recognized by evidence-based medicine, its role is to promote blood circulation, improve venous reflux and venous congestion, and increase range of motion, muscle strength, and joint stability, to accelerate the cartilage surface and synovial mesenchymal cell proliferation, and can stimulate the proliferation of cartilage cells around the lesion that support the degradation of cartilage regeneration; in KOA diagnosis and treatment, the application of artificial intelligence, computer gradually widely based on this, will be based on the movement of data mining the application result of rehabilitation therapy in the prevention and treatment of knee osteoarthritis, to provide theoretical basis for the prevention and treatment of knee osteoarthritis in China.

## 2. Materials and Methods

### 2.1. Case Source

A retrospective analysis was performed on 1612 KOA patients from the rheumatology department of our hospital from March 2016 to March 2020,including 893 males and 719 females, aged from 41 to 67 years, with an average age of (53.62 ± 7.81) years.

### 2.2. Diagnostic Criteria

Using the diagnostic criteria for knee osteoarthritis revised by the American College of Rheumatology [7]: (1) clinical symptoms: knee pain most of the time in the previous month; (2) X-ray showed osteophytes at the joint edge; (3) laboratory tests of arthritis were consistent with osteoarthritis; (4) age > 40 years; (5) morning stiffness < 30 min; (6) bone sound during joint movement; conforming to (1)+(2) or (1)+(3)+(5)+(6) or (1)+(4)+(5)+(6) can diagnose knee OA.

### 2.3. Inclusion and Exclusion Criteria

Inclusion criteria: (1) sufferers who met the above diagnostic criteria and diagnosed with knee osteoarthritis; (2) aged 40-70 years old; (3) all sufferers gave informed consent; (4) voluntarily accepted this study and insisted on completing the course of therapy.

Exclusion criteria: (1) sufferers with severe knee osteoarthritis, notoriously narrowed joint space, and surgical indications; (2) sufferers with knee OA with severe knee valgus or knee varus; (3) rheumatism, rheumatoid, and knee joint diseases such as gout, bone tuberculosis, and bone tumor; (4) sufferers with other diseases that seriously affect lower extremity function; (5) sufferers with severe heart, liver, kidney, and other organ diseases and blood diseases; (6) local skin infection, ulcers, or scars; (7) pregnant and lactating women.

Exclusion criteria: (1) subjects with poor compliance, complications, and unable to complete the entire course of therapy after inclusion; (2) those who do not meet the inclusion criteria; (3) those who cannot judge the efficacy or have incomplete data, which affect the judgment of efficacy.

### 2.4. Methods

#### 2.4.1. Intervention Methods

SQL Server management tool was used to retrieve the inpatient data from the database of the rheumatology department of our hospital, to extract and convert the data, establish the database according to the requirements, and lock the data after checking errors and cleaning noise data.

Data were collected including efficacy and immune factors of two groups: ImmunoglobulinA (IgA), ImmunoglobulinM (IgM), ImmunoglobulinG (IgG), complement C3, and complement C4; inflammatory indicators: erythrocyte sedimentation rate (ESR), serum interleukin receptor-7(IL-7R), tumor necrosis factor alpha (TNF-alpha), erythrocyte sedimentation rate (ESR), serum interleukin receptor-7(IL-7R), TNF-*α*, insulin-like growth factor (IGF), visual simulation scoring (VAS), Knee function score, Lysholm, and WOMAC; the relationship between VAS and Lysholm score and prognostic quality of life was analyzed. The recurrence of 12 months was compared between the two groups.

#### 2.4.2. Data Mining Methods

In this study, association analysis was used to find the correlation between the data of application effect of exercise rehabilitation therapy in the prevention and treatment of knee osteoarthritis. However, searching for correlation from large datasets may lead to lower efficiency, and the found correlation may be meaningless. Therefore, there are “support degree” and “confidence degree” in the research process. “Support degree” can delete those meaningless data based on grounds, while “confidence degree” can measure the possibility of setting rules. The main algorithms include Apriori algorithm, DHP algorithm, and DIC algorithm. Correlation analysis method to establish correlation pattern mining method, with the help of a variety of new optimization techniques, can effectively and efficiently reduce the application of exercise rehabilitation therapy in the prevention and treatment of knee osteoarthritis search space.

#### 2.4.3. Data Preprocessing

After treatment, effective was “F”; ineffective was “T”; VAS, IL-7R, TNF-*α*, IGF, IgA, IgM, IgG, C3, C4, WOMAC, and elevated were set as “T”; normal and decreased were set as “F”; Lysholm descending value is set as “T”; normal and rising value is set as “F.”

### 2.5. Statistical Methods

In this study, all the data were organized, and a corresponding database was established for it, and all the databases were entered into SPSS 26.0 for data processing, and the measurement data was tested for normality. The test between multiple sets is *F*, the independent sample *t* test is used for the data between sets, the paired sample *t* test is used for the data within the set, and the Mann–Whitney *U* test is not consistent with normality; the rate is expressed as %, and the test is *χ*^2^; sex; Kaplan-Meier test analyzed the cumulative readmission rate within one year; when *P* < 0.05, the disparity between the data was considered to be statistically extensive.

## 3. Results

### 3.1. Contrast of General Data

Using the data mining method, a total of 1612 sufferers were included. According to different therapy methods, they were divided into exercise rehabilitation therapy set (*n* = 786) and contrast therapy set (*n* = 826), as shown in Figure 1.

### 3.2. Contrast of Clinical Efficacy of the Two Therapy Methods in Sufferers

According to data mining, after therapy in different ways, there was a big disparity in the curative effect of the two therapy modes, mainly as the curative effect of the exercise rehabilitation therapy set was notoriously higher than that of the contrast therapy set (*P* < 0.05), as shown in Table 1.

### 3.3. Contrast of Joint Pain and Knee Function in Sufferers with Two Therapy Methods before and after Therapy

According to data mining, before therapy, VAS joint pain and Lysholm score were lower in both sets, and the disparity was not statistically extensive (*P* > 0.05). After therapy, VAS joint pain and Lysholm score in two sets were enhanced and exercised. The enhancement in the rehabilitation therapy set was notoriously better than that in the contrast therapy set (*P* < 0.05) (see Table 2).

### 3.4. Contrast of the Disparities in Laboratory Indicators before and after Therapy between the Two Sets of Sufferers with Different Therapy Methods

According to data mining, before therapy, there was no extensive disparity in laboratory serum inflammatory indexes and immune cytokines between the two sets (*P* > 0.05); after therapy, serum inflammatory indexes and immune cytokines in both sets were enhanced and exercised. The enhancement effect of the rehabilitation therapy set was notoriously better than that of the contrast therapy set (*P* < 0.05), as shown in Table 3 and Table 4.

### 3.5. Contrast of the Quality of Life of Sufferers with Different Therapy Methods in the Two Sets before and after Therapy

According to data mining, before therapy, the WOMAC scores of quality of life in both sets were higher, and the disparity was not statistically extensive (*P* > 0.05); after therapy, the WOMAC quality of life scores were enhanced in both sets, and the enhancement in the exercise rehabilitation therapy set was notoriously better than that in the contrast set (*P* < 0.05), as shown in Table 5.

### 3.6. Analysis of the Relationship between VAS and Lysholm Score and Prognosis Quality of Life

According to data mining, VAS, Lysholm score, and WOMAC score of prognosis quality of life were collected, and it was found that VAS score was notoriously positively correlated with WOMAC score (*r* = 0.579, *P* < 0.05); Lysholm score was notoriously positively correlated with WOMAC score (*r* = −0.563, *P* < 0.05) (see Figures 2 and 3).

### 3.7. Contrast of Recurrence within 1 Year between the Two Therapy Sets

According to data mining, the sufferers who completed the 12-month follow-up were recorded. During the follow-up period, 42 sufferers in the exercise rehabilitation therapy set were readmitted to the hospital for therapy, and the recurrence rate was 5.09%, which was notoriously lower than the 128 sufferers in the contrast therapy set, with a recurrence rate of 17.63%, and the disparity was statistically extensive. For academic significance (*χ*^2^ = 11.967, *P* < 0.05), see Figure 4.

## 4. Discussion

Modern medicine believes that the main pathological changes of KOA are articular cartilage degeneration, secondary bone hyperplasia and sclerosis, and subchondral bone cystic changes. However, the etiology and pathogenesis of KOA are not completely clear, and there is no effective therapy method [8]. Sports rehabilitation therapy breaks the traditional concept of rest therapy, is based on modern clinical fine anatomy, biomechanics, sports medicine, and rehabilitation medicine, focuses on scientific sports rehabilitation therapy, and focuses on the therapy of knee osteoarthritis [9]. However, there are few clinical application effects and situations of exercise rehabilitation therapy at present, and with the rapid development of the information age, the explosive growth of medical knowledge, and the continuous change of the disease spectrum, the clinical decision-making ability of doctors is facing severe challenges. Medication errors or misoperations caused by mistakes are one of the important causes of medical errors and even liability accidents [10]. Clinical decision support through massive objective reality data, medical guidance, literature, etc., with the help of computer's accurate and fast information storage, acquisition, and calculation capabilities, artificial intelligence technology, and computer logic, builds a knowledge base of various diseases and simulates the thinking of doctors in diagnosis and therapy It can provide doctors with intelligent classification, disease inquiry, differential diagnosis, rational drug use, therapy evaluation, and other services, effectively solve the limitations of doctors' knowledge, reduce human errors and omissions, and enhance the efficiency of drug use, thereby improving the level of medical care, service capabilities, and efficiency, reducing medical errors to bring beneficial help; on this basis, the application of artificial intelligence technology and intelligent therapy intelligence will provide powerful solutions [11]. Based on this, in order to explain the mechanism of exercise rehabilitation therapy in KOA from a clinical perspective and verify its effectiveness, this study will provide a simple and effective set of clinical recovery and clinical symptom enhancement after knee osteoarthritis therapy based on artificial intelligence data mining.

Among all kinds of rehabilitation therapy for arthritis, the role of exercise rehabilitation therapy is the most recognized by evidence-based medicine. Its functions promote blood circulation, enhance venous return and venous congestion, increase joint range of motion, muscle strength, and joint stability, promote the diffusion of synovial fluid to the cartilage surface and the intercellular substance, and can stimulate the proliferation of chondrocytes around the lesion area, supporting the regeneration of degenerated cartilage, and the strength of the sufferer's extensor muscles may increase the stability of the knee joint [12]. Clinical studies have shown that exercise rehabilitation is the most effective way to prevent and treat joint diseases and injuries and to support articular cartilage repair. Continuous passive movement of joints promotes the absorption of synovial fluid, which penetrates into articular cartilage, strengthens the metabolism of cartilage cells, and is beneficial to cartilage. The regeneration of functional quadriceps exercise in the therapy of knee osteoarthritis can effectively increase the stability of the knee joint and enhance the weight-bearing capacity of the knee joint [13]. The results of data mining showed that the therapeutic effect of the exercise rehabilitation group was significantly higher than that of the control group (*P* < 0.05).

In addition, data mining results showed that VAS pain and Lysholm score were improved in both groups after treatment, and the improvement in the exercise rehabilitation therapy group was significantly better than that in the control group (*P* < 0.05). The immune cytokines were enhanced, and the enhancement effect of the exercise rehabilitation therapy set was notoriously better than that of the contrast therapy set (*P* < 0.05); for sufferers who are unwilling to change behavior or have excessive pain and loss of joint function, KOA nondrug behavioral therapy is the first recommendation in terms of rehabilitation and prevention, while exercise rehabilitation therapy can enhance health-related symptoms and quality of life [14]. Physical rehabilitation is considered the basis for conservative disease management due to its extensive enhancement in sufferers with mild to severe KOA, whereas the main goals of exercise rehabilitation are pain relief, enhanced physiology, and effective participation in social activities, which can enhance physiological functions such as muscle strength, proprioception, range of motion, and cardiorespiratory function in sufferers with KOA to avoid abnormal body weight, mental status, and metabolism, as well as the risk of falling [15].

According to the data mining results, in this study, the sufferers who completed 12-month follow-up were recorded. During the follow-up period, 42 sufferers in the exercise rehabilitation therapy set were readmitted to the hospital for therapy, with a recurrence rate of 5.09%, which was notoriously lower than that in the contrast set of 128 sufferers, with a recurrence rate of 17.63%. There was statistical significance (*χ*^2^ = 11.967, *P* < 0.05). Physical rehabilitation therapy is a cost-effective and acceptable approach in the therapy and prevention of KOA, and the updated OA therapy guidelines of the American Society of Clinical Rheumatology strongly recommend that KOA sufferers participate in aerobic, resistance, and aquatic interventions, help enhance functional limitations in KOA sufferers, and reduce the risk of recurrence. Although KOA sufferers can use various forms of exercise rehabilitation therapy, due to the extensive impact of muscle strength on pain and lower limb function in KOA sufferers, lower limb strength training is an important component of most knee and hip osteoarthritis exercise rehabilitation therapy section [16]. The combination of muscle strength training and aerobic training helps to enhance symptoms in most sufferers with KOA, but the type of exercise should be selected based on an assessment of the individual sufferer's condition, and the range of motion should be increased due to the reduced range of motion in sufferers with KOA [17]. Sufferers with KOA also have impaired neuromuscular contrast and an increased risk of falls, so for sufferers, balance training should be part of the exercise regimen, and the sufferer's balance should be assessed at the start of training to ensure safe movement, which is often as part of an overall KOA exercise program, KOA sufferers with overweight problems should also manage their KOA symptoms through diet and weight management [18].

To sum up, this study is based on data mining; combined with information network technology, exercise rehabilitation therapy for KOA patients can effectively improve inflammatory and immune factors in patients, enhance knee joint function and prognosis quality of life, and reduce readmission rate, which is worthy of clinical application.

## Figures and Tables

**Figure 1:** Flow chart of data mining literature selection.

**Figure 2:** Analysis of the relationship between VAS and Lysholm scores and quality of life WOMAC score.

**Figure 3:** Analysis of the relationship between Lysholm score and prognosis quality of life WOMAC score.

**Figure 4:** Cumulative readmission of sufferers in the two sets within 1 year.

**Table 1:** contrast of clinical efficacy between the two sets of sufferers [*n* (%)].

Set	Effective	Efficient	Invalid	Total efficiency
Exercise rehabilitation therapy set (*n* = 826)	563 (68.16)	203 (24.58)	60 (7.26)	766 (92.74)
Contrast therapy set (*n* = 786)	355 (45.17)	292 (37.15)	139 (17.68)	647 (82.32)
*χ* ^2^				19.169
*P*				<0.001

**Table 2:** Contrast of joint pain and knee function in sufferers with two therapy methods before and after therapy ($\bar{x}\pm s$).

Set	VAS score		Lysholm score	
	Before therapy	After therapy	Before therapy	After therapy
Exercise rehabilitation therapy set (*n* = 826)	7.85 ± 1.06	1.26 ± 0.23^∗^	57.23 ± 8.51	87.63 ± 10.15^∗^
Contrast therapy set (*n* = 786)	7.57 ± 1.09	2.57 ± 0.69^∗^	57.63 ± 8.92	73.37 ± 9.81^∗^
*t*	0.352	-12.216	-0.562	6.326
*P*	0.572	<0.001	0.524	<0.001

Note: ^∗^ indicates that contrast with before therapy in this set, *P* < 0.05, the disparity is statistically extensive.

**Table 3:** Contrast of inflammatory factors before and after therapy in two sets of sufferers with different therapy methods.

Set	IL-7R (ng/L)		TNF-*α* (*μ*g/L)		IGF (*μ*g/L)	
	Before therapy	After therapy	Before therapy	After therapy	Before therapy	After therapy
Exercise rehabilitation therapy set (*n* = 826)	173.56 ± 63.53	140.46 ± 35.33^∗^	74.35 ± 18.56	50.69 ± 10.53^∗^	75.63 ± 31.59	53.69 ± 31.57^∗^
Contrast therapy set (*n* = 786)	173.93 ± 62.63	162.53 ± 39.57^∗^	73.35 ± 17.36	73.57 ± 13.39^∗^	74.69 ± 15.63	64.66 ± 14.65^∗^
*t*	0.359	-3.303	0.433	-4.958	0.416	-4.607
*P*	0.412	0.001	0.512	<0.001	0.537	<0.001

Note: ^∗^ indicates that contrast with before therapy in this set, *P* < 0.05, the disparity is statistically extensive.

**Table 4:** Immune factors and metabolic indexes before and after therapy in two sets of sufferers with different therapy methods.

Set	IgA (g/L)		IgM (g/L)		IgG (g/L)		C3 (g/L)		C4 (g/L)	
	Before therapy	After therapy	Before therapy	After therapy	Before therapy	After therapy	Before therapy	After therapy	Before therapy	After therapy
Exercise rehabilitation therapy set (*n* = 826)	2.39 ± 1.17	2.12 ± 0.91^∗^	1.19 ± 0.59	1.13 ± 0.52^∗^	12.56 ± 3.19	12.03 ± 2.02^∗^	113.25 ± 21.93	103.25 ± 19.47^∗^	26.89 ± 8.45	24.33 ± 6.42^∗^
Contrast therapy set (*n* = 786)	2.41 ± 1.16	2.30 ± 1.02^∗^	1.20 ± 0.84	1.16 ± 0.81^∗^	12.58 ± 3.26	12.56 ± 2.36^∗^	117.25 ± 22.63	113.52 ± 21.53^∗^	27.83 ± 9.41	25.96 ± 6.88^∗^
*t*	0.569	11.589	0.693	12.646	0.891	10.513	0.953	11.527	0.838	10.972
*P*	0.512	0.001	0.473	<0.001	0.305	<0.001	0.217	0.001	0.349	<0.001

Note: ^∗^ indicates that contrast with before therapy in this set, *P* < 0.05, the disparity is statistically extensive.

**Table 5:** Contrast of knee joint function and quality of life before therapy and after 1 month of therapy.

Set	WOMAC	
	Before therapy	After therapy
Exercise rehabilitation therapy set (*n* = 826)	66.37 ± 8.94	28.55 ± 4.89^∗^
Contrast therapy set (*n* = 786)	67.89 ± 9.46	47.56 ± 6.97^∗^
*t*	0.893	17.836
*P*	0.221	<0.001

Note: ^∗^ indicates that contrast with before therapy in this set, *P* < 0.05, the disparity is statistically extensive.

## Data Availability

The datasets used in this paper are available from the corresponding author upon request.
